# Developing Multiagent E-Learning System-Based Machine Learning and Feature Selection Techniques

**DOI:** 10.1155/2022/2941840

**Published:** 2022-01-30

**Authors:** Shrouk H. Hessen, Hatem M. Abdul-kader, Ayman E. Khedr, Rashed K. Salem

**Affiliations:** ^1^Faculty of Computers and Information, Menoufia University, Shebin Elkom, Egypt; ^2^Faculty of Computers and Artificial Intelligence, South Valley University, Hurghada, Egypt; ^3^Faculty of Computers and Information Technology, Future University in Egypt (FUE), Cairo, Egypt

## Abstract

Recently, artificial intelligence (AI) domain increased to contain finance, education, health, mining, and education. Artificial intelligence controls the performance of systems that use new technologies, especially in the education environment. The multiagent system (MAS) is considered an intelligent system to facilitate the e-learning process in the educational environment. MAS is used to make interaction easily among agents, which supports the use of feature selection. The feature selection methods are used to select the important and relevant features from the database that could help machine learning algorithms produce high performance. This paper aims to propose an effective and suitable system for multiagent-based machine learning algorithms and feature selection methods to enhance the e-learning process in the educational environment which predicts pass or fail results. The univariate and Extra Trees feature selection methods are used to select the essential attributes from the database. Five machine learning algorithms named Decision Tree (DT), Logistic Regression (LR), Random Forest (RF), Naive Bayes (NB), and K-nearest neighbors algorithm (KNN) are applied to all features and selected features. The results showed that the learning algorithm that has been measured by the Extra Trees method has achieved the highest performance depending on the evaluation of cross-validation and testing.

## 1. Introduction

During the last two years, global disasters have occurred, so all people are forced to use technologies to get their services remotely [1]. Technologies could allow users to achieve the appropriate task at a low cost and save time. Artificial intelligence (AI) is a trending topic in current days, which allows machine learning to be implemented for efficiency and performance [2]. Education, health, industry, and finance use artificial intelligence to develop their fields. Rapidly increasing education environment needs to use machine learning techniques which are considered one of the faces for AI [3].

Enhancing learning systems, especially e-learning systems in the educational process, has become necessary for the educational environment. Using an intelligent system is our target to organize the e-learning process. Continuous changes in the e-learning process led to emerging suitable techniques to deal with the requirements of students [4–6]. The e-learning system could allow students to use the benefits of this application anywhere, anytime. When using the e-learning system, there is a need to be supported by the multiagent model to cover the shortage of educational environment. Since many attributes are used in the e-learning process, multiagent is the best solution for the e-learning system. Agents could interact with others in the same environment, so the multiagent system could allow integration between agents [7, 8]. The multiagent system could allow e-learning attributes to interact and discover their relationship. In the e-learning system, students could use many features to enhance their performance [9]. Proposing the multiagent system could assist e-learning systems in improving various tasks for students. Using artificial intelligence systems is the way to enhance the performance of students by using feature selection methods [10, 11].

Machine learning algorithms are used to identify and predict the data to produce the best solution for a decision [3]. Machine learning algorithms are playing an essential role in different fields [12, 13] and especially in the field of education [14, 15]. Machine learning algorithms play an essential role in the educational process and feature selection algorithms. Feature selection algorithms could select only relevant features for high prediction by using various algorithms [16, 17]. Many feature selection algorithms could be used for efficiency, revealing irrelevant features.

This paper proposed an education system using multiagents to study interactive agents' effects to enhance e-learning. We integrated different agents: course, student, and different activities, and we applied different feature selection methods to select the most attributes that are playing an important role in enhancing the e-learning process. We applied five machine learning algorithms on selected features and evaluated ML algorithms' performance using different measurement methods to enhance the effect of the feature selection methods on the performance of the educational process.

In the next section, the literature review will illustrate the related work of predicting performance using machine learning algorithms and the features that affect the prediction of the education system.  Section 3 displays the main steps of the proposed system.  Section 4 discusses the results of applying ML algorithms on the selected features.  Section 5 provides a summary of the paper.

## 2. Related Works

Machine learning (ML) is an implementation part of artificial intelligence (AI) that enables the machine to learn from data to complete the task efficiently. It is considered a backbone of artificial intelligence approaches that are used to develop the prediction to enhance performance [2, 18].

Feature selection (FS) is considered important data before deploying machine learning algorithms [16, 17]. The feature selection could select only relevant and essential features from the data and ignore the redundant data [19]. Many researchers have used feature selection methods and machine learning algorithms to improve the educational process. For example, in [20], the authors proposed a learning system that implements a fuzzy methodology to detect the failure of students. The activity of students, subjects, and their background in education are the factors that affect performance. They used multicriteria of the fuzzy algorithm to get the rank of students which predict the score. The dataset consisted of 3 institutions that contained 131 students with 22 attributes.

In [21], the authors used machine learning algorithms to predict the performance of students in the faculty of Computer Science and Information Technology. They proposed supervised machine learning algorithms to predict the results of the examination so, they work under two steps. The preprocessing step is to prepare the data, clean it, and then use the machine learning algorithms to predict performance. They used several supervised algorithms, and the results proved that the logistic regression classifier gets the best results for 498 students.

In [22], the authors proposed a decision tree algorithm compared with the other three algorithms. They used Weka tools and test the data collected to predict failure and success. They tested the features that affect the accuracy based on the model results on gaining relevant features. The results of features selected five relevant features from ten total features. After using several popular machine learning algorithms (J48, Random Tree, and RepTree), they recommended that the decision tree algorithm is the best solution for high accuracy.

In [19], the authors proposed their study using feature selection in supervised machine learning algorithms for higher education. They used Weka mining tool in their experiments which is the most popular tool for mining. The dataset consists of 11 features that selected out 45 features to predict the student's residence country which was trained and tested with different methods. They used K-Fold, Hold-Out, and Leave One Out, and then the results found that Leave One Out obtained high accuracy with Random Forest, and GRAE algorithm results enhanced the accuracy and obtained the highest accuracy. In [23], the authors proposed a Generalized Feature Selection (GeFeS) method-based machine learning genetic algorithm to choose a subset of features that were unique and important. In this study, the method used an efficient and fast prediction method to optimize the performance for high accuracy and minimize the cost. Genetic Algorithm (GA) with the sequence of operators had been used to be more relevant and intelligent. Operators in GA are used to increase the capability which allows dealing with a variant dataset (small and large scale). This method succeeded in increasing the accuracy and evaluating F-measure, and then, the results were compared with other feature selection methods. The proposed algorithm could illustrate high performance compared with previous methods that were used before considering the same datasets. In [24], two feature selection methods are combined (CHI and MI) to measure the performance, which could evaluate the scores of features. The new features' scores had been normalized then, measuring the performance of the student in the education process as it considered important agent from the multiagent that were found in the educational sector. This study presented comparison results of using different predictive models and illustrated the accuracy for each model to develop the performance.

## 3. Methodology

The proposed multiagent framework-based e-learning educational system is shown in Figure 1. It consists of the following steps: data collection, preprocessing dataset, integrating dataset, feature extraction methods, splitting dataset, training and optimizing ML algorithms, and evaluating ML algorithms. We will describe each step as follows.

### 3.1. Data Collection

We used Open University Learning Analytics dataset [25] to make our experiment. This dataset contains seven multiagent described as CSV files, and each file contains a table with several features:

1. Courses: the courses that students should be studied per semester
2. Assessment of students: the results of all assessments should be submitted after being completed by students
3. Information about students: the student's basic information
4. Registration of students: the date that students are allowed to register for the course
5. Virtual learning environment of students: the interaction that belongs to students on each course could be recorded
6. Virtual learning environment: each material of courses could be found in different types and styles of learning; then, each student could access them and the activity of students could be recorded.
7. Assessment: the evaluation of students during the semester which contains the results of all assignments that had been submitted

The dataset includes many learning and activity types that could be applied for students in each course. The collected dataset evaluates the interaction that belongs to 32,593 students that interacted with 19 activity types and their styles in 22 courses. In our work, we will study the impact of using four agents that will be integrated named as follows: courses, students' information, virtual learning environment of students, and their VLE. These integrated agents will be illustrated to improve the learning system in the educational process. The following sections will describe the preprocessing steps on the dataset and propose a developed multiagent e-learning system that contains integrated four agents.  Table 1 describes each agent and its attributes.

### 3.2. Preprocessing Dataset

This paper tried to solve the problem by converting it into a binary classification problem. The student's info table includes a class label and the value of the class label contains four values: pass, fail, withdrawn, and distinction. The distinction is converted into a pass value and the withdrawn is converted into a fail value. We integrated the student's vle table with the VLE table into one table which is called student's learning style and activity; the names of learning and activities in the VLE table are extracted and added as attributes in the student's vle table and filling values of attributes by the number of total clicks for each student in a course.

### 3.3. Integrating Dataset

The integrated tables have been combined by using left join. The student's learning style and activity table is integrated with the student's info table which contains the following attributes “id student,” “code module,” and “code presentation” by implementing left join.

### 3.4. Feature Selection Methods

The key advantages of employing feature selection techniques are used to identify and select the most essential and most ranked features from the dataset. Machine learning algorithm-based feature selection methods are used to achieve the best performance. The two methods are used, namely, univariate and Extra Trees feature selection methods:

- Univariate feature selection is used to select the best features from all features depending on univariate statistical tests. In this method, each feature will have its own rank and score, and then, it is easy to select the high scored features considered as the best features.
- Extra Trees extended its function from the original set of the data sample. In the test set, each one of the test nodes with each one of the trees is supported with a number of random features depending on each one of the decision trees. Each decision tree should select the relevant feature-based mathematical algorithm [26, 27].

### 3.5. Splitting Dataset

The integrated dataset is partitioned into a training set of data and a testing set of data. The training set is used to optimize ML algorithms by implementing grid search and stratified cross-validation. Testing set is used to evaluate ML algorithms performance by four measurement methods: accuracy (A), precision (P), recall (R), and F-measure (F). The results of cross-validation and testing are registered for each ML algorithm.

### 3.6. Training and Optimizing ML Algorithms

Grid search with cross-validation is used to optimize ML algorithms and enhance the performance of algorithms. Grid search is a technique used for determining the best hyperparameters for ML algorithms in order to achieve the best results. CV splits the dataset into *k* subsets so that ML algorithms can be trained on k-1 subsets (the training set) andthe testing subsetis used to test machine learning algorithms. ML algorithms are used to develop a multiagent e-learning system. These algorithms are

1. Naive Bayes (NB) classifier is considered one of the classification supervised machine learning approaches assuming that there are two independent features. NB estimates relevant parameters, so it is considered one of the high classification techniques for relevant output [28].
2. Random Forest (RF) is a machine learning model used for classification problems that are used because of its flexibility. It could use to operate many decision trees at the first step of preprocessing data (training set step) and then calculate the average of prediction of the trees. Random Forest was used to estimate the accuracy in exploratory data analysis (EDA) step which could deal with large dataset. It is used as an effective way to deal with enormous features and retrieve estimated feature-based algorithm [29, 30].
3. Decision Tree (DT) classification supervised algorithm is the most popular algorithm for the machine learning algorithm. It has branches with nodes for constructing graphs to present internal node as test feature communicated in every leaf as result as gaining parent node, and then leaf could be assigned the label of the class. DT is classified as a top-down approach that starts from the root point of the tree. The branch is submitted as significance for its node to decide the label [28, 31]. Decision Tree Algorithm contains a root which splits into branches to make the prediction (decision) [28]. This algorithm is one of the most common algorithms that could address the problem in a process that identifies the solution accurately and fast.
4. Logistic Regression (LR) is one of the regression algorithms that play a part of prediction role and could develop the relationship among dependent variables and independent variables [32].

### 3.7. Evaluating ML Algorithms

There are many standard metrics used to evaluate ML algorithms called accuracy (A), precision (P), recall (R), and F-measure (F). True positive (TP), true negative (TF), false positive (FP), and false negative (FN) are defined as follows:

(1) $$\begin{array}{c} \text{accuracy}\left(A\right)=\frac{\text{TP}+\text{TN}}{\text{TP}+\text{FP}+\text{TN}+\text{FN}}, \end{array}$$

(2) $$\begin{array}{c} \text{precision}\left(P\right)=\frac{\text{TP}}{\text{TP }+\text{ FP}}, \end{array}$$

(3) $$\begin{array}{c} \text{recall}\left(R\right)=\frac{\text{TP}}{\text{TP}+\text{FN}}, \end{array}$$

(4) $$\begin{array}{c} F-\text{measure}\left(F\right)=\frac{2\cdot \text{precision}\cdot \text{recall}}{\text{precision}+\text{recall}}. \end{array}$$

## 4. Experiments and Results

### 4.1. Experiment Setup

This paper's experiments were run on Python 3. ML models were implemented using the sci-kit-learn package. ML algorithms are optimized using grid search with cross-validation. The dataset was partitioned into two parts: an 80% training set for optimizing models and registering cross-validation results and a 20% testing dataset (unseen data) for evaluating models and registering testing results. We conducted various experiments to study the effect of learning and activity types in the educational process using feature selection methods based on five ML algorithms: DT, KNN, NB, LR, and RF. First, feature selection methods have been applied to the database for determining the important features. Second, ML algorithms are used based on full features. Third, ML algorithms have been implemented on the top thirteen features that recorded the highest scores. Fourth, ML algorithms have been implemented as another experiment on the top six features that have the highest scores or rankings. The results of the cross-validation and testing have been recorded using accuracy (A), precision (P), recall (R), and F-measure (F).

### 4.2. Results of Applying Feature Selection Methods

In this section, we will describe the results of applying feature selection methods: univariate and Extra Trees on the database.

#### 4.2.1. Univariate Feature Selection Method

Univariate assigns scores for each feature, and we selected the important and best features based on high scores.  Table 2 shows the scores of all features of applying the univariate method on the dataset. We can see that the oucontent activity is registered that contains the first high score with 5494843.899. Forumng activity has registered the second high score with 3793119.894. Html activity has registered the lowest score at 1012.523433 for activities. Code presentation has registered the worst score at 0.377850061 for all features.

#### 4.2.2. Extra Trees Feature Selection Method

Extra Trees assigns ranking for each feature, and we selected the best features based on high ranking.  Figure 2 shows the ranking of all features of applying Extra Trees on the dataset. We can see that the homepage and quiz have the highest ranking at 12.5 and 12.24, respectively. The repeat activity has registered the lowest rank at 0.01. Resource, url, and code module have approximately the same rank at 6.78, 6.61, and 6.15, respectively.

### 4.3. Results of Applying ML Algorithms to Full Features

ML algorithms have been applied to full features, and the results of cross-validation and testing performance of applying ML algorithms have been recorded as shown in Table 3. In the cross-validation result, the RF has registered the highest performance (*A* = 88.14%, *P* = 88.51%, *R* = 88.12%, and *F* = 88.15%), while NB has recorded the lowest performance (*A* = 69.79%, *P* = 71.09%, *R* = 69.79%, and *F* = 68.89%). KNN has recorded the second-highest performance (*A* = 83.74%, *P* = 84.21%, *R* = 83.74%, and *F* = 83.74%). In the testing result, RF has registered the highest performance (*A* = 86.88%, *P* = 87.21%, *R* = 86.88%, and *F* = 86.89%), while NB has recorded the lowest performance (*A* = 69.44%, *P* = 70.72%, *R* = 69.44%, and *F* = 68.51%). KNN has recorded the second-highest performance (*A* = 82.23%, *P* = 82.51%, and *R* = 82.23%, *F* = 82.24%).

### 4.4. Results of Applying ML Algorithms to Thirteen Features

Two feature selection methods will be applied, thirteen features are selected because of their high ranking and scores. ML algorithms have been applied and the results of cross-validation and testing have been recorded.

#### 4.4.1. Thirteen Selected Features by Univariate

The top thirteen features, oucontent, forumng, quiz, homepage, subpage, ouwiki, resource, url, oucollaborate, glossary, dataplus, questionnaire, and externalquiz, have been selected. ML algorithms have been applied to thirteen features, and the results of cross-validation and testing performance of applying ML algorithms have been recorded as shown in Table 4.

In the cross-validation result, the RF has registered the highest performance (*A* = 86.5%, *P*=86.8%, *R* = 86.48%, and *F* = 86.55%), while NB has recorded the lowest performance (*A* = 66.19%, *P*=66.64%, *R* = 66.19%, and *F* = 65.52%). KNN has recorded the second-highest performance (*A* = 83.63%, *P*=84.11%, *R* = 83.63%, and *F* = 83.63%). In the testing result, RF has registered the highest performance (*A* = 85.72%, *P*=85.96%, *R* = 85.72%, and *F* = 85.73%), while NB has recorded the lowest performance (*A* = 65.19%, *P*=65.71%, *R* = 65.19%, and *F* = 64.37%). KNN has recorded the second-highest performance *A* = 82.32%, *P*=82.58%, *R* = 82.32%, and *F* = 82.33%.

#### 4.4.2. Thirteen Selected Features by Extra Trees

The top 13 features, homepage, quiz, oucontent, subpage, forumng, resource, url, code module, ouwiki, oucollaborate, page, questionnaire, and glossary with high ranking, have been selected. ML algorithms have been applied to 13 features, and the results of cross-validation and testing performance have been recorded as shown in Table 5.

In the cross-validation result, the RF has registered the highest performance (*A* = 87.6%, *P*=88.05%, *R* = 87.71%, and *F* = 87.7%), while NB has recorded the lowest performance (*A* = 68.82%, *P*=69.85%, *R* = 68.82%, and *F* = 67.98%). KNN has recorded the second-highest performance (*A* = 83.72%, *P*=84.2%, *R* = 83.72%, and *F* = 83.73%). In the testing performance, RF has registered the highest performance (*A* = 86.72%, *P*=87.08%, and *R* = 86.72%, *F* = 86.73%), while NB has recorded the lowest performance (*A* = 68.38%, *P*=69.52%, and *R* = 68.38%, and *F* = 67.45%).

### 4.5. Results of Applying ML Algorithms to Six Selected Features

After applying two feature selection methods, six features with high ranking or scores have been selected. ML algorithms have been applied and the results of cross-validation and testing have been recorded.

#### 4.5.1. Six Selected Features by Univariate

The top six features, oucontent, forumng, quiz, homepage, subpage, and ouwiki with high scores, have been selected. ML algorithms have been applied to six features, and the results of cross-validation and testing performance of applying ML algorithms have been recorded as shown in Table 6.

In the cross-validation result, the RF has registered the highest performance (*A* = 84.41%, *P*=84.71%, *R* = 84.38%, and *F* = 84.44%), while NB has recorded the lowest performance (*A* = 65.36%, *P*=65.78%, *R* = 65.36%, and *F* = 64.65%). KNN has recorded the second-highest performance (*A* = 83.38%, *P*=65.78%, *R* = 65.36%, and *F* = 64.65%). In testing, RF has registered the highest performance (*A* = 84.41%, *P*=84.71%, *R* = 84.41%, and *F* = 84.42%), while NB has recorded the lowest performance (*A* = 82.05%, *P*=82.35%, *R* = 64.01%, and *F* = 64.37%). KNN is recorded as the second-highest performance *A* = 82.32%, *P*=82.58%, and *R* = 82.05%, *F* = 82.07%).

#### 4.5.2. Six Selected Features by Extra Trees

The top six features, homepage, quiz, oucontent, subpage, forumng, and resource with high ranking, have been selected, and ML algorithms have been applied to six features, and the results of cross-validation and testing performance have been recorded as shown in Table 7.

In the cross-validation result, the RF has registered the highest performance (*A* = 85.5%, *P* = 85.81%, *R* = 85.48%, and *F* = 85.54%), while NB has recorded the lowest performance (*A* = 66.14%, *P* = 66.36%, *R* = 66.14%, and *F* = 65.66%). KNN has recorded the second-highest performance (*A* = 83.27%, *P* = 83.84%, *R* = 83.27%, and *F* = 83.73%). In the testing result, RF has registered the highest performance (*A* = 85.06%, *P* = 85.36%, *R* = 85.06%, and *F* = 85.08%), while NB has recorded the lowest performance (*A* = 65.52%, *P* = 65.68%, *R* = 65.52%, and *F* = 65.06%). KNN has recorded the second-highest performance (*A* = 82.16%, *P* = 82.54%, *R* = 82.16%, and *F* = 82.16%).

### 4.6. Discussion

Overall, the RF has achieved the highest performance for each experimental results.  Figure 3 displays the best model (RF) for 13 selected features. As can be seen, the RF has achieved the best performance using Extra Trees for cross-validation and testing (*A* = 87.6%, *P*=88.05%, *R* = 87.71%, and *F* = 87.7%) and (*A* = 86.72%, *P*=87.08%, *R* = 86.72%, and *F* = 86.73%), respectively.  Figure 4 displays the best model (RF) for 6 selected features. Moreover, the RF has achieved the highest performance using Extra Trees for cross-validation and testing (*A* = 85.5%, *P*=85.81%, *R* = 85.48%, and *F* = 85.54%) and (*A* = 85.06%, *P*=85.36%, *R* = 85.06%, and *F* = 85.08%), respectively.

## 5. Conclusion

This paper proposed a developed multiagent e-learning system to examine the interactions between agents that impact on e-learning process in the educational environment. The proposed framework briefly consists of the following steps: data collection, data preprocessing, integrating multiagents, feature extraction methods, and training and optimizing ML algorithms in addition to evaluating the performance of ML algorithms. In the integrating step, agents had been combined and used as tables named: course, student's info, student's vle, and VLE in one table using left join. In the feature selection steps, univariate and Extra Trees Classifier feature selection methods are used to select the most attributes that are relevant and play an important action in enhancing our multiagent framework. Different machine learning algorithms are used: DT, RF, LR, NB, and KNN, which are applied to select the high-ranked and relevant features. ML algorithms' performance was evaluated using different measurement methods: ACC, PER, REC, and FM. The results showed that RF with 13 selected features by Extra Trees has achieved the highest performance for cross-validation (ACC = 87.6%, PRE = 88.05%, REC = 87.71%, and FM = 87.7%) and testing (ACC = 86.72%, PRE = 87.08%, REC = 86.72%, and FM = 86.73%).

## Figures and Tables

**Figure 1:** The main steps of the proposed system.

**Figure 2:** All features rank by applying the Extra Trees feature selection method.

**Figure 3:** The best algorithms for 13 features.

**Figure 4:** The best algorithms for 6 features.

**Table 1:** Multiagent's features with data description.

Table/agent name	Column name	Data description
Student's info	Code module	The courses' names which students are allowed to register
	Code presentation	The name of the semester that students register for the course
	Id students	Unique numbers assigned to each student that is not repeated for another student
	Gender of students	Each student's gender (male or female)
	Region	The place where students live during studying the course
	Highest education	The latest level that students have before registering for the course
	IMD band	More specific places where students live during studying the course
	Age band	The interval of student's age
	Num of prev attempts	The number that students register for the course before
	Studied credits	The total credit hours of the courses for each student
	Disability	Disability for each student

Course	Code module	The name of each course
	Code presentation	The semester that each student registers for the course

Student's VLE	Code module	The name of the courses
	Code presentation	The semester name for each course that is assigned to students
	Id student	The number assigned to each student, and it must be unique
	Id site	The number that should be uniquely assigned to each material

VLE	Id site	The number assigned to each VLE material in the course
	Code module	The name of the course
	Code presentation	The semester that students studied the courses
	Activity types	The learning style of the courses that students studied in each semester

**Table 2:** All feature scores of applying univariate feature selection method.

Feature	Score
Oucontent	5494843.899
Forumng	3793119.894
Quiz	3080685.183
Homepage	2812271.074
Subpage	1098650.24
Ou wiki	519654.0067
Resource	307219.4371
Url	206070.6995
Oucollaborate	50797.46462
Glossary	45450.22849
Dataplus	44466.82491
Questionnaire	41164.68907
Externalquiz	19200.95953
Page	13807.02522
Ou elluminate	10236.97629
Dualpane	10128.68798
Folder	4052.247444
Html activity	1012.523433
Code module	41.73398396
Shared subpage	14.99873594
Repeat activity	2.253661372
Code presentation	0.377850061

**Table 3:** The results of cross-validation and testing by applying classifiers to full features.

Model	Cross-validation performance				Testing performance			
	A	P	R	F	A	P	R	F
DT	82.77	82.75	82.74	82.74	80.81	80.82	80.81	80.81
KNN	83.74	84.21	83.74	83.74	82.23	82.51	82.23	82.24
**NB**	**69.79**	**71.09**	**69.79**	**68.89**	**69.44**	**70.72**	**69.44**	**68.51**
LR	80.4	80.5	80.4	80.34	80.34	80.39	80.34	80.28
**RF**	**88.14**	**88.51**	**88.12**	**88.15**	**86.88**	**87.21**	**86.88**	**86.89**

The highest values and low values are represented as bold values.

**Table 4:** The results of cross-validation and testing for applying classifiers on 13 features by univariate.

Model	Cross-validation performance				Testing performance			
	A	P	R	F	A	P	R	F
DT	80.42	80.38	80.4	80.4	78.76	78.76	78.76	78.76
KNN	83.63	84.11	83.63	83.63	82.32	82.58	82.32	82.33
**NB**	**66.19**	**66.64**	**66.19**	**65.52**	**65.19**	**65.71**	**65.19**	**64.37**
LR	78.89	79.0	78.89	78.85	79.33	79.36	79.33	79.32
**RF**	**86.5**	**86.8**	**86.48**	**86.55**	**85.72**	**85.96**	**85.72**	**85.73**

The highest values and low values are represented as bold values.

**Table 5:** The results of cross-validation and testing for applying ML algorithms to thirteen features by Extra Trees.

Model	Cross-validation performance				Testing performance			
	A	P	R	F	A	P	R	F
DT	82.24	82.26	82.1	82.23	82.24	82.26	82.1	82.23
KNN	83.72	84.2	83.72	83.73	82.25	82.53	82.25	82.26
**NB**	**68.82**	**69.85**	**68.82**	**67.98**	**68.38**	**69.52**	**68.38**	**67.45**
LR	80.04	80.04	80.04	80.01	80.6	80.59	80.6	80.59
**RF**	**87.6**	**88.05**	**87.71**	**87.7**	**86.72**	**87.08**	**86.72**	**86.73**

The highest values and low values are represented as bold values.

**Table 6:** The results of cross-validation and testing for applying classifiers on six features by univariate.

Models	Cross-validation performance				Testing performance			
	A	P	R	F	A	P	R	F
DT	78.04	78.06	78.06	78.0	77.84	77.84	77.84	77.84
KNN	83.38	83.87	83.38	83.38	82.05	82.35	82.05	82.07
**NB**	**65.36**	**65.78**	**65.36**	**64.65**	**64.01**	**64.6**	**64.01**	**62.98**
LR	77.49	78.12	77.49	77.2	78.44	79.0	78.44	78.2
**RF**	**84.41**	**84.71**	**84.38**	**84.44**	**84.41**	**84.71**	**84.41**	**84.42**

The highest values and low values are represented as bold values.

**Table 7:** The results of cross-validation and testing of applying classifiers to 6 selected features by Extra Trees.

Model	Cross-validation performance				Testing performance			
	A	P	R	F	A	P	R	F
DT	78.05	78.06	78.08	78.1	77.97	77.97	77.97	77.97
KNN	83.27	83.84	83.27	83.27	82.16	82.54	82.16	82.16
**NB**	**66.14**	**66.36**	**66.14**	**65.66**	**65.52**	**65.68**	**65.52**	**65.06**
LR	78.26	78.67	78.26	78.07	78.58	79.0	78.58	78.39
**RF**	**85.5**	**85.81**	**85.48**	**85.54**	**85.06**	**85.36**	**85.06**	**85.08**

## Data Availability

Open University Learning Analytics dataset is downloaded from https://www.kaggle.com/rocki37/open-university-learning-analytics-dataset.
